The article "Application of an Artificial Intelligence System Recognition Based on the Deep Neural Network Algorithm" was published in 2022. Journal: Comput Intell Neurosci.

# Application of an Artificial Intelligence System Recognition Based on the Deep Neural Network Algorithm

**DOI:** 10.1155/2022/4623188

**Published:** 2022-07-14

**Authors:** Yaru Zhang, Qian Zhang, Jingxuan Yang

**Affiliations:** ^1^College of Electrical Information, Langfang Normal University, Langfang, China; ^2^College of Math and Physics, Langfang Normal University, Langfang, China

## Abstract

With the development of artificial intelligence and computer technology, the deep neural network algorithm is applied to the intelligentization of various fields of production and life. However, from the current application status, the application of artificial intelligence technology has many shortcomings. Based on this, this paper starts with the deep neural network algorithm, takes face recognition as the research tool, and deeply studies how to use the deep neural network algorithm to demonstrate the application of intelligent face recognition in complex environments. A face recognition neural network algorithm is proposed, and the accuracy of the algorithm is checked by testing. The results show that the average accuracy of a single sample in the LFW dataset is 99.17%, and the efficiency of using a single sample is close to that of many smelting models, which can be applied to various intelligent recognition scenarios.

## 1. Introduction

Artificial intelligence recognition technology refers to a research and technology that uses computers and intelligent platforms. Artificial intelligence recognition technology can identify reality and simulate various human thoughts and behaviors, creating intelligent automated systems through intelligence and technology. As an automatic, intelligent, and scientific computer technology, computer artificial intelligence recognition technology can accurately identify, scientifically judge and simulate human thinking patterns from abstraction to concreteness, and finally fully reflect it through computer programs. Computer artificial intelligence identification technology is widely used in various fields. Compared with other computer technologies, artificial intelligence identification technology has a broader application prospect and can provide humans with more efficient, convenient, and high-quality services. In the application process, computer technical analysis techniques can detect and analyze the affected data. For example, the scanning tool used in supermarkets is a smart tool. Through the analysis of the product barcode, relevant information such as product quality, unit price, name, etc., is fully revealed. Sellers can calculate the total price by entering the quantity. As always, computers are used to develop machine knowledge [1]. In addition, computer technology knowledge can also be used in industrial office automation, production intelligence, etc. This is necessary to improve many aspects of human performance and performance levels. Computer artificial intelligence technology has a certain high-end nature. Using the existing functions of computers, it can effectively simulate human thinking and consciousness, and truly reflect human thinking with the help of computer programs. Compared with other computer technologies, the future development space of computer artificial intelligence recognition technology is broader. In-depth research and analysis of the application of computer artificial intelligence recognition technology has certain practical significance. Based on the research of automation technology, intelligence, and computer technology, artificial intelligence computer technology realizes real-time, decision-making research and simulation by thinking about human reasoning, from abstraction to concreteness, and finally through computer programs. Computer technology intelligent analysis technology has been widely used in many fields. Information technology covers a wider range than other technologies and can provide better, more comfortable, and better services for human beings. Therefore, starting from the deep neural network algorithm, intelligent face recognition technology has always been a research topic, and in-depth analysis of how deep face recognition algorithms use deep neural network algorithms in complex environments [2]. In the 1940s, scientists invented a neuron abstract model according to the structure of neurons. The model includes the functions of input, calculation, processing, and output, as shown in Figure 1.

The article "Application of an Artificial Intelligence System Recognition Based on the Deep Neural Network Algorithm" was published in 2022. Journal: Comput Intell Neurosci.

## 2. Literature Review

Face recognition technology has made great progress after the deep learning theory was put forward. Hazra used a layer-by-layer greedy algorithm to make up for the difficult problem of multi-layer neural network training, improve the computing ability of the computer, and quickly carry out deep neural network training through GPU, which has attracted extensive attention of many scholars [3]. Yang designed a Deep Face Recognition System (DeepFace) as a deep neural network. The accuracy rate of the LWF face database is above 97%, and the effect is good [4]. He improved the deep learning algorithm [5]. Aziz proposed the DeepID algorithm [6]. The test accuracy of the LFW face database is 97.5%, and the test accuracy of the LFW face database based on the improved DeepID2 algorithm is 99.2%. Duan used the Gabor feature algorithm to extract edge features through linear filtering, expression, and action on face recognition [7]. Since then, facenet proposed by Chandrika uses the triple loss function to extract the feature information of a human face and applies it to the process of biometric recognition and clustering. The accuracy of the face database (LWF) reached 99.63% [8]. Since then, major Internet companies have made considerable progress through unremitting efforts. Maleki, E. and others have also made great achievements in face recognition research [9]. In 2017, Alipay launched the brush payment function for the first time and achieved the separation of human-machine and the payment. At the same time, “face-swiping payment” was also rated as one of the top 10 technologies in the world by MIT Technology Review in 2017; someone proposed a deep convolutional neural network-based in-depth study of superhuman faces, which simultaneously recognizes facial discovery, integration, various functions of head body estimation, and gender awareness. Experiments show that the algorithm can capture international and local data in faces, and better improve deep learning performance. Liu, H. based on the improvement of L-SoftMax proposed angular SoftMax (A-SoftMax) to learn face discrimination features. It imposes a discrimination constraint on the hypersphere manifold, which is essentially located on the same manifold as the prior knowledge of the face [10]. The recognition results on the LFW/YTF/MegaFace face library are better than the previous loss functions; face recognition is based on large interval cosine loss (2018). It provides an improved bead cosine loss function for deeper face recognition. Normalizing and improving the cosine decision limits are more effective in increasing and decreasing class differences. This paper summarizes the loss function in the face recognition model from SoftMax to CosFace, and puts forward ArcFace with an angle margin method in the loss function, which obtains more recognizable depth features. An ensemble new end-to-end convolutional neural network model for face detection is being prepared. Super-resolution and refinement networks are used to produce realistic and clear images, showing the separation of faces and faces separately; this addresses the low face solution seen in unrestricted situations.

The article "Application of an Artificial Intelligence System Recognition Based on the Deep Neural Network Algorithm" was published in 2022. Journal: Comput Intell Neurosci.

When extracting local features, the method of image segmentation is often used. Some scholars propose to cut the image horizontally into several copies. Then the final feature is to integrate all local features. However, this method can only be applied to the highly aligned pictures of pedestrians; otherwise, it may lead to the dislocation of local features of the head and other parts between pedestrians; thus, it is of little significance in comparison. Alignedreid makes relevant improvements based on the above deficiencies and has made great progress. In the real shooting scene, it is difficult to ensure that the proportion of pedestrians in the picture can be consistent, i.e., when shooting pedestrians, it may be close-up or long-range. When cutting the image to extract local features, an automatic alignment model based on the SP distance is used to align the local features of pedestrians by calculating the shortest distance, such that there will not be too much error in the final verification.

## 3. Method

### 3.1. Face Recognition Algorithm

AdaBoost is a redesigned algorithm; its main idea is to introduce multiple weak classifiers for the same dataset. The weak classifiers are then combined into a strong classifier, and several power classifiers are concatenated into the final cascaded classifier to distribute the dataset [11].

#### 3.1.1. Characterizing Picture Features

The Haar feature is the basis of the AdaBoost algorithm; it is the rectangular feature of the input picture. As shown in Figure 2, rectangular features mainly include two rectangles, three rectangles, and four rectangles, which correspond to edge features, linear features, and specific direction features, respectively. Different rectangular features can be selected to represent different regional features of the face [12].

#### 3.1.2. Finding Eigenvalues from Integral Graph

After the face features are represented by rectangular features, the eigenvalues should be obtained through the integral graph. Here, the integral graph is equivalent to an accelerator because when training the classifier, the appropriate Haar feature is selected to represent the corresponding facial region, which can be selected only after continuous arrangement and combination of different rectangular features. The integral graph is equivalent to an accelerator [13]. For example, a 24 × 24 window can produce at least 100000 features, and the amount of calculation to obtain these eigenvalues is very large. The advantage of an integral graph is that it can traverse the picture once to obtain the pixel values of different regions, which greatly simplifies the calculation of eigenvalues as shown in Equation fd1:

(1) $$\begin{array}{c} ij\left(i,j\right)=\sum_{k\leq i,l\leq j}f\left(m,l\right). \end{array}$$

Integral graph siv algorithm:

S (*i*, *j*) is used to represent numbers in sentences. The beginning is represented by the following equation:

(2) $$\begin{array}{c} s\left(k,-1\right)=0. \end{array}$$

Let *ij* (*i*,*j*) represent an image, as shown in the following equation:

(3) $$\begin{array}{c} ij\left(-1,i\right)=0. \end{array}$$

Scan line by line and recursively compute the sum *s* (*i*, *j*), and the value of the image *ij* (*i*, *j*) in the row direction of each pixel (*i, j*) is as shown in the following equation:

(4) $$\begin{array}{c} s\left(i,j\right)=s\left(i,j-1\right)+f\left(i,j\right);ii\left(i,j\right)=ii\left(i-1,j\right)+s\left(i,j\right). \end{array}$$

The article "Application of an Artificial Intelligence System Recognition Based on the Deep Neural Network Algorithm" was published in 2022. Journal: Comput Intell Neurosci.

#### 3.1.3. Constructing Weak Classifier

After selecting the number of rectangles and the value of, you need to perform visual impairment training for each *f*, as shown in the following equation:

(5) $$\begin{array}{c} k\left(x,f,p,\theta \right)=\left\{\begin{array}{c} \begin{array}{cc} 1, & pf\left(x\right)<p\theta , \end{array}\\ \begin{array}{cc} 0, & \text{else.} \end{array} \end{array}\right. \end{array}$$

During training, start to calculate the number of eigenvalues of the current element and the eigenvalues of the previous element, and calculate the weight of all positive samples, which is represented by *T*+; the weight of all negative parameters is represented by T−; the weight of all good models before this season is represented by *S*+; the weights of all negative samples before the current season are represented by S-; and the initial error distribution after that is shown in the following equation:

(6) $$\begin{array}{c} r=\min\left[S^{+}+\left(T^{-}-S^{-}\right),S^{-}+\left(T^{+}-S^{+}\right)\right]. \end{array}$$

The minimum classification error is an optimal weak classifier.

#### 3.1.4. Cascade Strong Classifier

After *T* iterations, *T* optimal weak classifiers are obtained, and a strong classifier can be combined in the following ways, as shown in the following equation:

(7) $$\begin{array}{c} C\left(x\right)=\left\{\begin{array}{c} \begin{array}{cc} 1, & \sum_{t=1}^{T}\alpha_{t}h_{t}\left(x\right)\geq \frac{1}{2}\sum_{t=1}^{T}\alpha_{t} \end{array}\\ \begin{array}{cc} 0, & \text{else}, \end{array} \end{array}\right. \end{array}$$

As shown in the following equation:

(8) $$\begin{array}{c} \alpha_{t}=\log\frac{1}{\beta_{t}}=\text{Log}\frac{1-\varepsilon_{t}}{\varepsilon_{t}}. \end{array}$$

Completing the cascade of strong classifiers is the ultimate goal of the AdaBoost algorithm. In the classification calculation, first input all the face images, then select a good weak classifier, use the Haar feature to detect the images in multiple regions and scales, and output a large number of sub-window images to the input images. These sub-windows are continuously classified when passing through each weak classifier. As long as positive samples are found, they will automatically enter the next level classifier for screening until the screening of the whole cascade classifier is completed [14]. The operation flow diagram is shown in Figure 3.

The article "Application of an Artificial Intelligence System Recognition Based on the Deep Neural Network Algorithm" was published in 2022. Journal: Comput Intell Neurosci.

### 3.2. Face Intelligent Calibration

#### 3.2.1. Face Feature Point Location Algorithm Based on CLNF

CLNF is a new patch structure with local neural fields (LNFs), leading to the study of nonlinear dependencies of pixel density and feature point alignment probability. CLNF also uses the frequency conversion of the point to change the reliability of the area [15].

Furthermore, the LNF field model can obtain the relationship between pixels (adjacent and distant) by studying the similarity and volatility of distances. Each element of the LNF geographic model has a different area of interest.

#### 3.2.2. Training and Fitting of the CLNF Model

During model training, all parameters are jointly optimized, focusing on the model parameters, as shown in the following equation:

(9) $$\begin{array}{c} \alpha =\left\{\alpha_{1},\alpha_{2},...,\alpha_{K1}\right\},\\ \theta =\left\{\theta_{1},\theta_{2},...,\theta_{K1}\right\},\\ \beta =\left\{\beta_{1},\beta_{2},...,\beta_{K1}\right\},\\ \gamma =\left\{\gamma_{1},\gamma_{2},...,\gamma_{K1}\right\}. \end{array}$$

Give *M* blocks, as shown in the following equation:

(10) $$\begin{array}{c} {\left\{x^{\left(q\right)},y^{\left(q\right)}\right\}}_{q=1}^{M}. \end{array}$$

The above formula is the training data, in which each *x*^(*q*)^ is shown in the following equation:

(11) $$\begin{array}{c} x^{\left(q\right)}=\left\{m_{1}{}^{\left(q\right)},m_{2}{}^{\left(q\right)},...,m_{n}{}^{\left(q\right)}\right\}. \end{array}$$

The above formula is an input sequence (pixel value in the possible region of feature points), as shown in the following equation:

(12) $$\begin{array}{c} y^{\left(q\right)}=\left\{y_{1}^{\left(q\right)},y_{2}^{\left(q\right)},...,y_{n}^{\left(q\right)}\right\}. \end{array}$$

The above formula is a real value output sequence.

During training, select the value to maximize the conditional log likelihood of LNF on the training sequence, as shown in the following equations:

(13) $$\begin{array}{c} L\left(\alpha ,\beta ,\theta ,\gamma \right)=\sum_{q=1}^{M}\log\;P\left(m^{\left(q\right)}|x^{\left(q\right)}\right), \end{array}$$

(14) $$\begin{array}{c} \left(\bar{\alpha },\bar{\beta },\bar{\gamma },\bar{\theta }\right)=\underset{\alpha ,\beta ,\gamma ,\theta }{\arg\max}\left(L\left(\alpha ,\beta ,\gamma ,\theta \right)\right). \end{array}$$

Through the derivation of the partial differential equation of formula (13), (13) is transformed into a multivariate Gaussian form, as shown in the following equations:

(15) $$\begin{array}{c} P\left(y|x\right)=\frac{1}{{\left(2\pi \right)}^{\left(n/2\right)}{\left|\sum \right|}^{1/2}}\exp\;{\left(-\frac{1}{2}y-\mu \right)}^{T}\sum^{-1}\left(m-\mu \right), \end{array}$$

(16) $$\begin{array}{c} \sum^{-1}=2\left(A+B+C\right). \end{array}$$

The article "Application of an Artificial Intelligence System Recognition Based on the Deep Neural Network Algorithm" was published in 2022. Journal: Comput Intell Neurosci.

## 4. Results and Analysis

Tests are performed on Multi-Pie face packets. Photos of 200 people were selected for the experiment. The experiments compared the CLNF results with the normalized data model (AAM) and the local model limit (CLM) as shown in Table 1 [16].

Through the in-depth study of face detection and face calibration, the principle and detection steps of the AdaBoost face detection algorithm are described in detail. From the test results, the algorithm can accurately determine the front and side of the image. The CLNF facial feature point localization algorithm is deeply researched. Local neural models have been shown to capture nonlinear relationships between pixel values and outputs, and CLNF algorithms have been studied and tested. Experimental results show that the algorithm can recognize face points in real time. The study of this algorithm will preprocess the image input of the deep convolutional network model [17].

The goal of face recognition is to judge who the face belongs to. The purpose of face verification is to verify whether two faces belong to the same person; the face detection and recognition system is based on intelligent video analysis, and automatically analyzes and recognizes video image information without manual intervention, recognizes existing faces, and timely detects the intrusion of strangers in the monitoring area, in the fastest and best way. It carries out early warning, effectively assists management personnel to deal with it, and minimizes false alarms and omissions; at the same time, you can also view on-site video, which is convenient for post-event management and inquiries, which is a more basic work than face recognition. We can W transform the face recognition problem into a face verification problem. The simplest idea is that the process of one face recognition is to carry out multiple face verifications, verify with different individuals one by one, and finally determine the individual corresponding to the face [18]. The flow of face verification is shown in Figure 4. It can be *w* refined into H steps of face feature extraction, feature dimensionality reduction, and feature matching classification. Feature extraction represents the face as a feature vector. Feature matching uses a classifier to compare the similarity of two vectors and judge whether they belong to the same person. Firstly, we introduce the algorithm of extracting face feature vector with deep convolution neural network, and then introduce the algorithm of feature dimensionality reduction and feature matching [19].

The article "Application of an Artificial Intelligence System Recognition Based on the Deep Neural Network Algorithm" was published in 2022. Journal: Comput Intell Neurosci.

In order to derive face vector properties using foldable neural networks, it is found that the last layer of the network is the entire connection layer, and the product of the connection process can be used as the input image.

The DeepID network is a face-to-face training network provided by the Chinese University of Hong Kong. It is a network representative specializing in face recognition. Each face image is represented as a vector of 160 parts during the connection process, and the output of the electrical device is 97.45% compared to other products. Faces in the LFW dataset [20] are proven. The entire network process uses the product of the 4th convolutional layer and the 3rd pooling layer as the concatenated input. It is determined that the higher the level of the CNN, the greater the similarity in understanding, and we can learn both local and international features [21].

Connect the DeepID layer to SoftMax for classification, and regard the training process as a problem of human face classification rather than face verification. The dimension of the DeepID layer should be much smaller than that of the input layer, i.e., the classification quantity, such that the full connection unit sending one layer can fully learn the information of different categories, so as to better distinguish the categories with DeepID.

Then, with these five key points as the center, cut from the face-aligned image with three different sizes, and finally generate the hungry subgraph [22]. The upper part represents the 10 face regions obtained by clipping, including five global subgraphs on the left and five local subgraphs with five key points on the right. The lower part of the graph represents *h* scales of different sizes. At the same time, the image is divided into gray image and color image, and 10 × 3 × 2 = 60 face patches are obtained. For a face image, a total of 60 patches are obtained to train a convolutional neural network model. Each network can obtain 160 dimensional features. At the same time, after a patch is horizontally flipped, 160 dimensional features can also be obtained through the convolution neural network model corresponding to the horizontal flipping. These features can be spliced to obtain a 160 × 60 × 2 = 19200 dimensional feature vector [23]. Although the features obtained by one model are only 160 dimensions, we can obtain higher dimensional feature vectors by training multiple patch models, so as to better represent the face image.

In the neural network, the main function of the function is to reduce the structural capacity of the network; thus, W, usually the activation function, is a nonlinear function. In normal neural networks, the sigmoid function or the TA address function is usually used to simulate neuron function [24]. In convolutional neural networks, the modified linear unit (ReLu) is often used more. The basic principle of deep learning is based on an artificial neural network. The signal enters from one neuron, passes through a nonlinear activation function, and is passed to the next layer of neurons; then, through the activation of the layer of neurons, it continues to pass down, and so on. This repeats until the output layer. It is precisely because of the repeated superposition of these nonlinear functions that the neural network has enough capacity to capture complex patterns and achieve state-of-the-art results in various fields. Obviously, the activate function plays an important role in deep learning and is also one of the active research areas. ReLu is also the reason for the great success of the deep neural network. The advantages of ReLu are mainly reflected in two aspects: avoiding the problem of gradient dissipation and making the network sparse [25].

The article "Application of an Artificial Intelligence System Recognition Based on the Deep Neural Network Algorithm" was published in 2022. Journal: Comput Intell Neurosci.

When we train the convolutional neural network, we use a model similar to VGGNeT. Unlike the input size of 224 × 224 used by VGGNeT, we use the input size of 100, which makes the parameters of the whole model less and can be trained on a GPU with smaller video memory. The network structure of the model is shown in Table 2:

There are 10 layers of taxation and 5 layers of taxation, a total of 15 layers. In each convolutional layer, we use a convolutional kernel of size 3 and delay 1 to control the same input and output images for each convolutional layer. In the first four pooling layers, we use Maxpooling, which can *w* halve the size of the image passing through this layer. In the last pooling layer, we used AVGpooling led average on a point of a large 7 × 7 image, and appended 320 feature maps, equivalent to a 320-dimensional vector. We use this 320-dimensional vector to represent the feature vector of the face. To avoid overfitting, we added the release process after this vector and set the release to 0.4. Then, there is an n-dimensional full connection layer. After each convolution layer except cohv52 layer, we added a nonlinear activation function, namely ReLu function or its variant. Because the result of the poo coincidence of cohv52 is the feature vector representing the face, we hope this vector is dense and fully contains information; thus, we did not add the activation function after cohv52 [26].

Therefore, we would like to provide more models as trained models. The patches centered on the left eye, right eye/left mouth corner, and right mouth also correspond to the left, right, left, and right parts of the first image. If the original image size is 100 x 100, cut out four squares from the center of the original image with a size of 50 × 50.

The article "Application of an Artificial Intelligence System Recognition Based on the Deep Neural Network Algorithm" was published in 2022. Journal: Comput Intell Neurosci.

The role of pool2 layer is also to convert the image input as 50×50 into the image output as 25 × 25. Its function is to reduce the image size without changing the image range. We consider replacing the pool2 layer operation with the image clipping operation, i.e., clipping the input 50 × 50 image into four smart *x* smart images. Unlike the operation of pool2 layer, it has four outputs and changes the range of images, and the four images do not overlap each other. With left mouth corner and right mouth corner as the center, for each patch, we will connect the network structure from conv21 layer to FC6 in Table 2. In this way, a 320-dimensional vector can be obtained for each patch, and a loss function can be calculated respectively. In the training process, we add the four sub-loss functions to obtain the loss function of the whole model for training. The network structure of the new model is shown in Table 3. The convolution process of each of the four training cores is equivalent to the convolution process of their respective training cores at the same time. In addition, we cut the patch during the training process to avoid the preprocessing work of cutting the patch before training. This model not only uses the information of the original image, but also uses the patch information of the key points of the four faces. Therefore, we call this model the key point model based on the key points of the face.

We train the convolutional neural network on GPU and joint Bayesian training on CPU. The deep learning training framework used is CAFFE, which adopts the data parallel method for parallel training on four GPUs of a machine. The experimental environment is shown in Table 4.

We use a cascade classifier based on the face detection algorithm. For face key point detection, we use a face key point detection algorithm based on cascaded convolutional neural networks. For facial coordination, we modeled the H point of the left eye, right eye, and nose to make a face that can be tilted at the same angle. Through face-to-face communication, we obtain face-to-face images of size 100 x 100 based on our understanding of the deep neural network training or experiments.

Through the convolutional neural network model, we get 320 cross-sectional feature vectors to represent the face. This feature vector can be reduced to a lower space for better data before entering the classifier on the proof surface. After reducing the size, we demonstrate better accuracy on the LFW dataset. First, we compare a model and use the PCA size reduction method to compare the accuracy of the image vector reduction to variance rather than the LFW length. The results are shown in Table 5. As can be seen, reducing the size to a smaller size (108–280) achieves higher accuracy. If the size is too small, the result will be worse due to data loss. In the subsequent experiments, we performed the first reduction for the characteristics of a model.

The article "Application of an Artificial Intelligence System Recognition Based on the Deep Neural Network Algorithm" was published in 2022. Journal: Comput Intell Neurosci.

For the feature vectors of two faces, we can judge whether they belong to the same person by Euclidean distance or joint Bayesian method. We compare the accuracy of the two methods on LFW. To improve efficiency, we use vector features obtained from different convolutional neural network models and divide them in two ways. Experimental results show that Bayesian ion fusion is more effective than directly applying Euclidean in face analysis because it uses category data from the training data. The result is shown in Figure 5.

## 5. Conclusion

This paper studies the application of deep convolutional neural networks in facial recognition. The main points are as follows:

1. This paper summarizes the influencing factors of face recognition effect, and puts forward the main problems to enhance the generalization of the algorithm.
2. The AdaBoost face detection algorithm and the CLNF feature point location algorithm are analyzed and studied. The CLNF algorithm is trained using multi pie face databases and tested in the actual scene. The results show that the algorithm can accurately locate face feature points.
3. The structure of the 34 layer residual network is improved using the global convolution layer instead of the global average pooling layer, which solves the problem that adding padding during multiple convolution and pooling operations will cause the effective receptive field of the pixels in the center region of the final feature map to be larger than that of the pixels in the edge region. The improved network is trained by the CASIA-WebFace face database and the face recognition model is obtained. The test of the LFW database shows that the accuracy of the improved model reaches 98.3% and increases by 2.2%.
4. In the improved network, by splicing the depth residual equivalent mapping module, the equivalent mapping of side face and front face in-depth space is realized. The front face in the LFW database is partially deleted and the proportion of side face in the test sample is increased. The test shows that the accuracy of side face recognition by the network model has reached 94.3% and increased by 7%.
5. According to the residual learning theory, three different network structure models are designed, including a 28-layer and two 56-layer network structures. Using the CASIA-WebFace face database and the LFW database, the three designed network structure models and the 34-layer network model are compared. The results show that the 28-layer residual network model is a small model, has short training time, and little difference in the recognition accuracy compared with the other three models. In the actual scene test, the 28-layer residual network model stitching the dream module is better than not stitching the dream module. The network model can effectively reduce the Euclidean distance between the side face and the front face, and enhance the generalization of the algorithm for side face recognition.
6. According to the residual learning theory, three different network structure models are designed, including a 28-layer and two 56-layer network structures. Three network structure models and the 34-layer network model are compared and verified using the CASIA-WebFace face database and the LFW database. The results show that the 28-layer residual network model is a small model, has short training time, and little difference in the recognition accuracy compared with the other three models. In the actual scene test, the 28-layer residual network model splices the dream module rather than the dream module. The network model effectively reduces the Euclidean distance between the side face and the front face, and enhances the generalization of the algorithm for side face recognition.

The article "Application of an Artificial Intelligence System Recognition Based on the Deep Neural Network Algorithm" was published in 2022. Journal: Comput Intell Neurosci.

Practice has proved that the application of intelligent analysis based on deep neural network algorithms is possible, which effectively improves the intelligence degree of some industries, meets the needs of the development of artificial intelligence in all walks of life, makes up for the lack of intelligent industrial transformation in traditional industries, and improves the degree of social intelligence and industrial development.

## Figures and Tables

**Figure 1:** Neuron model.

**Figure 2:** Rectangular features.

**Figure 3:** Operation flow chart of the AdaBoost algorithm.

**Figure 4:** Face verification process.

**Figure 5:** Comparison of the Euclidean distance and joint Bayesian effect (broken line).

**Table 1:** Comparison of the test results.

Positioning method	Average error (%)	Accuracy (%)
AAM	4.83	94.56
CLM	3.71	98.22
CLNF	1.42	99.16

**Table 2:** Model network structure.

Layer name	Type	Nuclear size	Interval	Output size
Transform 11	Dispute	3 × 3	1	100 × 100 × 32
Transform 12	Dispute	3 × 3	1	100 × 100 × 64
Pool1	Max pooling	2 × 2	2	50 × 50 × 64
Transform 21	Dispute	3 × 3	1	50 × 50 × 64
Transform 22	Dispute	3 × 3	1	50 × 50 × 128
pool2	Max pooling	2 × 2	2	25 × 25 × 128
Transform 31	Dispute	3 × 3	1	25 × 25 × 96
Transform 32	Dispute	3 × 3	1	25 × 25 × 192
Pool3	Max pooling	2 × 2	2	13 × 13 × 192
Transform 41	Dispute	3 × 3	1	13 × 13 × 128
Transform 42	Dispute	3 × 3	1	13 × 13 × 256
Pool4	Max pooling	2 × 2	2	7 × 7 × 256
Transform 51	Dispute	3 × 3	1	7 × 7 × 160
Transform 52	Dispute	3 × 3	1	7 × 7 × 320
pool5	Avg pooling	7 × 7	1	1 × 1 × 320
Dropout	Dropout			1 × 1 × 320
fc6	Fully dispute			N

The article "Application of an Artificial Intelligence System Recognition Based on the Deep Neural Network Algorithm" was published in 2022. Journal: Comput Intell Neurosci.

**Table 3:** Model structure based on the key point position of the human face.

Layer name	Type	Nuclear size	Interval	Output size
Transform 11	Dispute	3 × 3	1	100 × 100 × 32
Transform 12	Dispute	3 × 3	1	100 × 100 × 64
Pool1	Max pooling	2 × 2	2	50 × 50 × 64
Transform 21	Dispute	3 × 3	1	50 × 50 × 64
Transform 22	Dispute	3 × 3	1	50 × 50 × 128
Slice	Slice	-	-	(25 × 25 × 128) × 4
Transform 31	Dispute	3 × 3	1	(25 × 25 × 48) × 4
Transform 32	Dispute	3×3	1	(25 × 25 × 96) × 4
Pool3	Max pooling	2 × 2	2	(13 × 13 × 96) × 4
Transform 41	Dispute	3 × 3	1	(13 × 13 × 64) × 4
Transform 42	Dispute	3 × 3	1	(13 × 13 × 128) × 4
Pool4	Max pooling	2 × 2	2	(7 × 7 × 128) × 4
Transform 51	Dispute	3 × 3	1	(7 × 7 × 80) × 4
Transform 52	Dispute	3 × 3	1	(7 × 7 × 160) × 4
dropout5	Dropout			(7 × 7 × 160) × 4
fc5	Fully dispute			160 × 4

**Table 4:** Experimental environment.

Operating system	RedHat 6.4
CPU	Intel xeon CPU E5-2620 v2 @ 2.10 GHz
GPU	Nvidia Tesla K20 m,5G video memory
Memory	32G

**Table 5:** Comparison of the dimension reduction effects of PCA.

Dimensionality reduction	LFW accuracy
No PCA	0.9760
PCA 50	0.9613
PCA 100	0.9755
PCA 150	0.9765
PCA 180	0.9772
PCA 200	0.9765
PCA 250	0.9782
PCA 280	0.9782
PCA 300	0.9778

## Data Availability

The data used to support the findings of the study are included within the article.
